# GHK Peptide Inhibits Bleomycin-Induced Pulmonary Fibrosis in Mice by Suppressing TGFβ1/Smad-Mediated Epithelial-to-Mesenchymal Transition

**DOI:** 10.3389/fphar.2017.00904

**Published:** 2017-12-12

**Authors:** Xiao-Ming Zhou, Gui-Liang Wang, Xiao-Bo Wang, Li Liu, Qin Zhang, Yan Yin, Qiu-Yue Wang, Jian Kang, Gang Hou

**Affiliations:** ^1^Department of Respiratory Medicine, Shengjing Hospital of China Medical University, Shenyang, China; ^2^Department of Respiratory and Critical Care Medicine, The First Hospital of China Medical University, Shenyang, China

**Keywords:** GHK, TGF-β1, pulmonary fibrosis, epithelial-to-mesenchymal transition, Smad, collagen

## Abstract

**Objective:** Idiopathic pulmonary fibrosis is an irreversible and progressive fibrotic lung disease that leads to declines in pulmonary function and, eventually, respiratory failure and has no effective treatment. Gly-His-Lys (GHK) is a tripeptide involved in the processes of tissue regeneration and wound healing and has significant inhibitory effects on transforming growth factor (TGF)-β1 secretion. The effect of GHK on fibrogenesis in pulmonary fibrosis and the exact underlying mechanism have not been studied previously. Thus, this study investigated the effects of GHK on bleomycin (BLM)-induced fibrosis and identified the pathway that is potentially responsible for these effects.

**Methods:** Intratracheal injections of 3 mg/kg BLM were administered to induce pulmonary fibrosis in C57BL/6 mice. GHK was administered intraperitoneally at doses of 2.6, 26, and 260 μg/ml/day every other day from the 4th to the 21st day after BLM instillation. Three weeks after BLM instillation, pulmonary injury and pulmonary fibrosis was evaluated by the hematoxylin-eosin (HE) and Masson’s trichrome (MT) staining. Chronic inflammation index was used for the histological assessments by two pathologists blindly to each other. Tumor necrosis factor (TNF)-α and IL-6 levels in BALF and myeloperoxidase (MPO) activity in lung extracts were measured. For the pulmonary fibrosis evaluation, the fibrosis index calculated based on MT staining, collagen deposition and active TGF-β1 expression detected by ELISA, and the expression of TGF-β1, α-smooth muscle actin (SMA), fibronectin, MMP-9, and TIMP-1 by western blotting. The epithelial mesenchymal transition index, E-cadherin, and vimentin was also detected by western blot. The statistical analysis was performed by one-way ANOVA and the comparison between different groups were performed.

**Results:** Treatment with GHK at all three doses reduced inflammatory cell infiltration and interstitial thickness and attenuated BLM-induced pulmonary fibrosis in mice. GHK treatment significantly improved collagen deposition, and MMP-9/TIMP-1 imbalances in lung tissue and also reduced TNF-α, IL-6 expression in bronchoalveolar lavage fluid (BALF) and MPO in lung extracts. Furthermore, GHK reversed BLM-induced increases in TGF-β1, p-Smad2, p-Smad-3 and insulin-like growth factor-1 (IGF-1) expression.

**Conclusion:** GHK inhibits BLM-induced fibrosis progression, the inflammatory response and EMT via the TGF-β1/Smad 2/3 and IGF-1 pathway. Thus, GHK may be a potential treatment for pulmonary fibrosis.

## Introduction

Idiopathic pulmonary fibrosis (IPF) is a severe respiratory disease characterized by progressive and diffuse pulmonary fibrosis and restrictive ventilation dysfunction that eventually leads to respiratory failure. Given that pulmonary fibrosis is characterized by a progressive pulmonary functional decline (Behr, 2013), studies seeking safe and effective treatments for pulmonary fibrosis are a crucial priority. TGF-β1 is known to play a key role in the pathogenesis of pulmonary fibrosis by activating Smad signaling pathways (Hu et al., 2003; Stolzenburg et al., 2016), and interventions targeting TGF-β1 or Smad signaling pathways are widely believed to have potential as treatments for pulmonary fibrosis (Stolzenburg et al., 2016).

Gly-His-Lys (GHK) is a tripeptide with an amino acid sequence of glycyl-histidyl-lysine and is a normal component of human plasma (Pickart and Thaler, 1973). GHK levels reflect regenerative capacity, and GHK plays an important role in tissue remodeling processes (Pickart, 2008)—wound healing and skin remodeling—induced by the stimulation of collagen and glycosaminoglycan synthesis and breakdown (Wegrowski et al., 1992). As a very important regulator of the wound healing process, TGF-β interacts with dermal fibroblasts and participates in various aspects of fibrogenesis, including the production of extracellular products, such as collagens, the EMT and the inflammatory process (Shinde and Frangogiannis, 2014; Moustakas and Heldin, 2016; Walton et al., 2017). It has been revealed that GHK has significant inhibitory effects on TGF-β1 secretion *in vitro* and *in vivo* (Border et al., 1992; Isaka et al., 1996; Simeon et al., 2000; Arul et al., 2005; Gruchlik et al., 2014). It has also been shown that fibroblasts derived from patients with COPD were responsible for impaired collagen remodeling leading to MMP/TIMP imbalances. Moreover, GHK was also reported to decrease the gene expression of IGF-1 (Pickart et al., 2014), which stimulates TGF-β1 transcription and protein expression in dermal fibroblasts *in vitro* (Ghahary et al., 1998). Therefore, confirming the hypothesis that GHK inhibits the TGF-β1/Smads pathway may provide new insights into the means by which pulmonary fibrosis can be treated. However, to date, no study has examined the effects of GHK on pulmonary fibrosis. Thus, to test the above hypothesis, we established a pulmonary fibrosis mouse model through BLM instillation and explored the therapeutic effects of GHK on BLM-induced pulmonary fibrosis in the mouse model. In addition, we elucidated the mechanisms underlying the protective effects of GHK against pulmonary fibrosis.

## Materials and Methods

### Animals

Specific pathogen-free male C57BL/6 mice were purchased from Liaoning Changsheng Biotechnology Company (Benxi, China) and were maintained under controlled conditions (indoor temperature: 22 ± 1°C and humidity: 40 ∼ 60%) and a 12-h dark-light cycle. The mice were fed standard laboratory chow and water. All animal experiments were approved by the Institutional Animal Care and Use Committee of China Medical University and performed in accordance to the Guide for the Care and Use of Laboratory Animals (Ministry of Science and Technology of China, 2006) and the related ethical regulations of our university. Our Guide for the Care and Use of Laboratory Animals meets United States regulations which are according to the Assessment and Accreditation of Laboratory Animal Care International (AAALAC) accreditation.

### BLM-Induced Pulmonary Fibrosis in Mice

Fifty male C57BL/6 mice aged eight to 9 weeks and weighing 18–22 g were randomly divided into the following five experimental groups (*n* = 10 per group): (I) a normal control group, (II) a BLM group, (III) a BLM+2.6 μg/ml/day GHK group, (IV) a BLM+26 μg/ml/day GHK group and (V) a BLM+260 μg/ml/day GHK group. The mice were anesthetized with 300 mg/kg chloral hydrate and were intratracheally injected with 3 mg/kg BLM (Meilun Biotechnology Co., Ltd., Dalian, China) in 100 μl of saline via tracheostomy to induce pulmonary fibrosis. The mice in the control group received an intratracheal injection of the same volume of vehicle (saline). The BLM+GHK groups received GHK (with a purity > 95%, China Peptides Co., Ltd., Shanghai, China) in 500 μl of PBS intraperitoneally (i.p.) every other day from the 4th to the 21st day after BLM instillation. The mice in the control group received PBS i.p. every other day. The doses of GHK used herein were based on data regarding the concentration of the drug in human plasma (Pickart and Thaler, 1973; Arul et al., 2007) and the results of a previous study (Park et al., 2016).

The mice were sacrificed on 21st day after the intratracheal administration of BLM or saline. Following sacrifice, the lung tissues were rapidly excised. Some of the left lungs were fixed in 4% paraformaldehyde for HE and MT staining. Other left lungs were used for the harvesting of BALF, which was performed by lavaging the left lung three times with 500 μl of saline via a tracheal catheter, while additional left lungs were weighed (wet weight). The BALF supernatants were stored at -80°C for protein detection. Some of the right lungs were harvested and stored at -80°C for subsequent analysis by real time quantitative polymerase chain reaction (qPCR) and western blotting, while other right lungs were perfused with cryomatrix (Thermo, New York, NY, United States) for immunofluorescence staining.

### Lung Myeloperoxidase (MPO) Activity in Lung Extracts

To measure MPO activity, we homogenized the right lungs in 50 mmol/L PBS containing 0.5% hexadecylammonium bromide and 5 mmol/L EDTA (pH = 6.0). After the lung extracts were centrifuged at 12500 *g* for 20 min at 4°C, the supernatants were incubated in 50 mmol/L PBS containing 30% H_2_O_2_ and *o*-dianisidine dihydrochloride (167 μg/ml, Sigma–Aldrich, St. Louis, MO, United States). Enzymatic activity was determined spectrophotometrically by measuring the change in absorbance at 460 nm over 3 min (Rittirsch et al., 2008).

### Enzyme-Linked Immunosorbent Assay (ELISA)

Active TGF-β1 expression was measured using an ELISA kit (Boster, Wuhan, China), according to the manufacturer’s instructions. After the reaction, the optical density (OD) was measured at 450 nm by a microplate reader (Roche Molecular Diagnostics, Light Cycler 480II, Carlsbad, CA, United States).

In addition, collagen expression was measured with a Sirius Red Total Collagen Detection Kit (Chondex, #9062, Redmond, WA, United States), according to the manufacturer’s instructions, using 1 mg of tissue per mouse. The optical density was measured at a wavelength of 500 nm.

Tumor necrosis factor (TNF)-α and IL-6 levels in BALF were determined using the appropriate mouse ELISA kits (Mouse TNF-α ELISA MAX Deluxe Set and Mouse IL-6 ELISA MAX Deluxe Set, BioLegend, San Diego, CA, United States).

### Histologic Analysis

#### HE and MT Staining

Lung tissues were fixed in 4% paraformaldehyde for 24 h, dehydrated in an ethanol gradient, and embedded in paraffin. Successive 5-μm lung sections were placed on slides and subjected to HE and MT staining, according to previously described methods, with minor modifications (Arul et al., 2007; Hou et al., 2015). Pulmonary fibrosis severity was quantified by calculating the MT staining pulmonary collagen-positive area (blue) using Image-Pro Plus 6.0 software (Media Cybernetics, Silver Spring, MD, United States). The lung sections were graded by two independent pathologists (Yuan Miao, and Qianze Dong, Associated Professors of Pathology, China Medical University) to determine fibrosis severity using the scale shown below, as described in previous studies (Gwinn et al., 2011). The pathologist determined (1) a severity score for fibrosis and chronic inflammation and (2) the distribution (% area affected) of fibrosis or chronic inflammation in the lung section. The fibrosis score was evaluated by MT with the following scale: 0 = within normal limits, 1 = minimal fibrosis (thin, wispy fibrils), 2 = mild fibrosis (small areas of fibril coalescence), 3 = moderate fibrosis (larger areas of more solid collagen deposition), and 4 = marked and severe fibrosis. The distribution of fibrosis was assessed by semi-quantitatively determining the percentage of the entire lung section that was affected by fibrosis. The severity index was calculated as follows: severity index = severity score (0 ∼ 4) × % area affected (0 ∼ 100%/100). Each score was determined by two observers blinded to the treatment groups who examined between 4 and 16 fields in all lung lobes (depending on the size and homogeneity of the histological changes) using light microscopy (200× magnification). The mean difference of the evaluation results by two independent pathologists has been calculated.

### Western Blot Analysis

Lung tissues were homogenized in ice-cold radioimmuno precipitation (RIPA) lysis buffer (Beyotime Institute of Biotechnology, Haimen, China). After the lung extracts were centrifuged (12,000 × *g*, 10 min at 4°C), the supernatant was collected, and protein concentrations were determined using a Bicinchoninic Acid (BCA) Protein Assay Kit (Beyotime Institute of Biotechnology). Bovine serum albumin was used as the standard. Equal amounts of protein (40 μg) were separated by 7.5 ∼ 12% SDS-PAGE and then transferred electrophoretically onto polyvinylidene difluoride (PVDF) membranes (Millipore, Bedford, MA, United States). The blotted membranes were blocked with 5% non-fat dry milk (w/v) in Tris-buffered saline with 0.1% Tween-20 (TBS-T) for 1 h at room temperature and then incubated with the following primary antibodies overnight at 4°C: anti-Smad2 (1:1,000 dilution, Cell Signaling Technology), anti-phospho-Smad2 (1:1,000 dilution, Cell Signaling Technology), anti-Smad3 (1:1,000 dilution, Cell Signaling Technology), anti-phospho-Smad3 (1:1,000 dilution, Cell Signaling Technology), anti-TGF-β1 (1:1000 dilution, Abcam), anti-IGF-1 (1:500 dilution, Abcam), TIMP-1 (1:500 dilution, Santa Cruz), MMP-9 (1:1000 dilution, R&D), fibronectin (1:500 dilution, Santa Cruz), E-cadherin (1:2000 dilution, CST), vimentin (1:2000 dilution, CST), and α-SMA (1:2000 dilution, CST). After being rinsed thrice with TBS-T at 5-min intervals, the membranes were incubated with horseradish peroxidase-labeled goat anti-rabbit IgG (1:2000 dilution; Biosynthesis Biotechnology Co., Ltd., Beijing, China) or goat anti-mouse IgG (1:2,000 dilution; Biosynthesis Biotechnology Co., Ltd., Beijing, China) for 1 h. These secondary antibodies and an enhanced chemiluminescence (ECL) kit (GE Healthcare, United States) were applied to generate chemiluminescent signals. All western blotting data are from experiments performed in triplicate. Densitometry analysis was performed using ImageJ6.0 software (National Institutes of Health, Bethesda, MD, United States).

### Quantitative Reverse Transcriptase Polymerase Chain Reaction (qRT-PCR) for TGF-β1 mRNA

Total RNA was extracted from frozen lung tissues with TRIzol reagent (TaKaRa Biotechnology Co., Ltd., Dalian, China) and was reverse-transcribed using a reverse transcription kit (TaKaRa Biotechnology Co., Ltd., Dalian, China). The resulting cDNA was used as a template for quantitative RT-PCR, which was performed with primers specific for TGF-β1 and β-actin (see in **Table 1**), according to the instructions for the SYBR Premix EX Taq Kit (TaKaRa Biotechnology Co., Ltd.), and a 7900HT Fast Real-Time PCR System (Applied Biosystems, Foster City, CA, United States).

**Table 1:** Nucleotide sequences of primers used for PCR.

Gene		Primer Sequence (5′–3′)
TGFβ1	Forward	CAACAATTCCTGGCGTTACCT
	Reverse	CGAAAGCCCTGTATTCCGTCT
β-actin	Forward	CCAGAGCAAGAGAGGTATCCTGAC
	Reverse	TTGTAGAAGGTGTGGTGCCAGAT


### Immunofluorescence Staining

For immunostaining, frozen sections (5 μm) were prepared (Frozen Section Medium Neg-50; Richard-Allan Scientific, Kalamazoo, MI, United States), fixed with cold acetone for 2 min, dried and then stored at -80°C. The sections were subsequently blocked with PBS+5% normal goat serum and 0.3% Triton X100 for 60 min, after which they were treated with primary antibodies specific for E-cadherin [E-Cadherin (4A2) Mouse mAb 1:50; 14472, Cell Signaling Technology, Danvers, MA, United States) in a humidified chamber overnight at -4°C. Detection was achieved with compatible Alexa Fluor fluorescein-conjugated secondary antibodies (Invitrogen, Carlsbad, CA, United States). The nuclei were counterstained with DAPI and covered with ProLong Gold antifade reagent with DAPI (Life Technologies Corporation, OR, United States). The preparations were analyzed with an Olympus BX53fluorescence microscope (Olympus, Tokyo, Japan), and the images were captured with Cellsens Dimension Life Science Imaging Software (Olympus, Kyoto, Japan).

### Statistical Analysis

All data are presented as the mean ± SEM. Data were analyzed by one-way ANOVA using SPSS 17.0 (SPSS Institute Inc., Chicago, IL, United States). Comparisons between two groups were evaluated by an unpaired Student’s *t*-test. *p* < 0.05 was considered statistically significant.

## Results

### GHK Attenuated BLM-Induced Pulmonary Fibrosis in Mice

One-time intratracheal treatment with BLM led to a significant increase in the lung W/D weight ratio and weight loss in mice (**Figures 1A,B**). However, the weight loss and the increase in the W/D weight ratio caused by BLM instillation were remarkably reversed by GHK treatment. MPO activity was assessed in lung tissue extracts to determine the inflammation level in the lung (**Figure 1C**). BLM instillation led to an increase in MPO levels in the BLM group compared with the control group, whereas GHK treatment significantly reduced MPO levels in the GHK treatment groups compared with the BLM group. On the 21st day after BLM stimulation, we performed HE (**Figures 1D,E**) and MT staining (**Figure 2**) to assess the above mentioned histopathological changes and lung tissue fibrosis. We noted clear morphologic changes, including apparent increases in inter-alveolar septal thickness, alveolar destruction, and inflammatory cell infiltration of the interstitium, in lung tissues treated with BLM; however, treatment with GHK at all three doses reduced inflammatory cell infiltration and interstitial thickness and attenuated BLM-induced pulmonary fibrosis in mice. Beside the inflammatory changes in pathological evaluation, we also evaluated the inflammatory cytokine expression in BALF. It is found that GHK could reduce the increased TNF-α and IL-6 levels in bleomycin-induced lung injury (**Figures 1F,G**). MT staining was used to assess collagen deposition in the pulmonary interstitium (**Figure 2**). Lungs treated with BLM intratracheally displayed large amounts of collagen deposition compared with control lungs. However, GHK treatment reduced collagen deposition and preserved lung architecture. The tissue sections were evaluated by assessments of chronic inflammation severity and fibrosis severity, as well as quantification of distribution areas. Analysis of the chronic inflammation index and the fibrosis index showed that GHK treatment significantly attenuated chronic inflammation and fibrosis. We used a Sirius Red Collagen Kit to quantify total collagen deposition in lung tissue and showed that BLM instillation increased total collagen deposition in the lung, results consistent with the Masson’s staining results; however, GHK treatment attenuated BLM-induced collagen deposition, indicating that GHK attenuated BLM-induced pulmonary fibrosis.

**FIGURE 1:** Effects of GHK on lung histological changes in mice with BLM-induced fibrosis. **(A)** BLM administration caused significant body weight loss, while GHK treatment attenuated body weight loss. **(B)** The lung W/D weight ratio was calculated using some left lobes. BLM administration increased the W/D weight ratio, whereas GHK reversed the change caused by BLM administration. **(C)** MPO activity levels in lung extracts. BLM administration increased MPO activity in the lung extracts, while GHK treatment normalized MPO activity in the lung extracts. **(D)** Chronic inflammation was significantly induced by intratracheal BLM administration, while GHK treatment reduced BLM-induced chronic inflammation. **(E)** Lung sections were stained with HE for histological assessment, and representative images are shown. **(F)** TNF-α levels in BALF were evaluated by ELISA kits. **(G)** IL-6 levels in BALF were evaluated by ELISA kits. The bars represent the mean ± SEM; statistical analysis was performed by one-way ANOVA and Turkey’s multiple-comparison test; compared with control group, ^##^*P* < 0.01; compared with BLM group, ^∗^*P* < 0.05, ^∗∗^*P* < 0.01.

**FIGURE 2:** Effects of GHK treatment on BLM-induced collagen deposition and assessments of fibrosis severity in mice. **(A)** Lung sections were stained with MT and then numerically scored for fibrosis severity and distribution. Representative photomicrographs showing the severity scores of the different groups are shown. **(B)** The fibrosis index was calculated with the severity score as follows: (0 ∼ 4) × % area affected (0 ∼ 100%)/100. **(C)** The lung sections were graded by two independent pathologists blinded to the treatment groups. The mean calculation of the difference of fibrosis severity index by the two individual pathologists has been shown. **(D)** Total collagen in lung tissue was detected by a Sirius Red Total Collagen Detection Kit. BLM increased collagen deposition in lungs of mice, whereas GHK treatment decreased collagen deposition in lung tissues. The bars represent the mean ± SEM values; statistical analysis was performed by one-way ANOVA and Turkey’s multiple-comparison test; compared with control group, ^##^*P* < 0.01; compared with BLM group, ^∗^*P* < 0.05, ^∗∗^*P* < 0.01.

### GHK Restores TIMP-1/MMP-9 Balance in BLM-Induced Fibrosis

Increases in the expression of MMP-9, which is also known as gelatinse A, may lead to degradation of all the components of the extracellular matrix and numerous non-matrix proteins in pulmonary fibrosis. Increases in the expression of TIMP-1, an inhibitor of MMP-9, lead to the resolution of pulmonary fibrosis. Thus, we detected MMP-9 and TIMP-1 protein expression in lung tissue in BLM-induced fibrosis (**Figure 3**). MMP-9 levels were remarkably increased, while TIMP-1 levels were decreased in the BLM group compared with the control group. Treatment with GHK attenuated this imbalance in pulmonary fibrosis.

**FIGURE 3:** GHK treatment restored the TIMP-1/MMP-9 balance in BLM-induced fibrosis in mice. **(A)** TIMP-1 and MMP-9 protein expression, as measured by western blot analysis, in lung tissues in each group. **(B,C)** The densitometry values for the proteins were normalized to those of β-actin. All data represent the mean ± SEM of three independent experiments performed in triplicate. Statistical analysis was performed by one-way ANOVA and Turkey’s multiple-comparison test; compared with control group, ^##^*P* < 0.01; compared with BLM group, ^∗^*P* < 0.05, ^∗∗^*P* < 0.01.

### GHK Suppresses BLM-Induced EMT in Pulmonary Fibrosis in Mice

The conversion of epithelial cells into mesenchymal cells, also known as EMT, is one of the crucial processes in pulmonary fibrosis. In this study, we detected the expression of the classic EMT markers E-cadherin, vimentin, fibronectin, and α-SMA in the lung tissues of mice (**Figure 4**). The results showed that the mRNA and protein expression levels of the epithelial marker E-cadherin were decreased in the BLM group compared with the control group, whereas the protein expression levels of the mesenchymal markers vimentin, fibronectin, and α-SMA were significantly increased in the BLM group compared with the control group. Treatment with GHK suppressed EMT and reversed the changes in the expression of E-cadherin, vimentin, fibronectin and α-SMA. The trends in E-cadherin expression in the lung sections of the mice in each group that were demonstrated by immunofluorescence staining (**Figure 4C**) were similar to those demonstrated by western blotting.

**FIGURE 4:** Effects of GHK on BLM-mediated EMT in mice with BLM-induced fibrosis. **(A)** Fibronectin, E-cadherin, vimentin, and α-SMA protein expression, as measured by western blot analysis, in lung tissues in each group. **(B)** The densitometry values for the proteins were normalized to those of β-actin. **(C)** Immunofluorescence staining was performed to detect E-cadherin protein expression (green) in lung tissue sections in each group. The nuclei were stained by DAPI (blue). Representative images of each group are shown. All data represent the mean ± SEM of three independent experiments performed in triplicate. Statistical analysis was performed by one-way ANOVA and Turkey’s multiple-comparison test; compared with control group, ^##^*P* < 0.01; compared with BLM group, ^∗^*P* < 0.05, ^∗∗^*P* < 0.01.

### GHK Alleviates Pulmonary Fibrosis via the TGF-β1/Smad2/3 Signaling Pathway in BLM-Induced Pulmonary Fibrosis

To determine whether GHK exerts its anti-fibrotic effects by inhibiting TGF-β1, a potent profibrotic factor, in BLM-induced IPF, we evaluated TGF-β1 protein and mRNA levels in lung tissue by western blotting and real time qPCR, respectively. In addition, we also measured TGF-β1 activity in lung tissue. BLM instillation significantly increased TGF-β1 protein expression and activity in lung tissue, changes that were reversed by GHK in a dose-dependent manner (**Figure 5**). TGF-β1 mRNA levels were measured by quantitative real-time PCR in each group. TGF-β1 mRNA levels were markedly increased in the BLM group compared with the control group. GHK decreased TGF-β1 mRNA levels in a dose-dependent manner in BLM-induced pulmonary fibrosis in mice (**Figure 5A**).

**FIGURE 5:** Effects of GHK on TGF-β1 mRNA and protein expression in mice with BLM-induced fibrosis. **(A)** TGF-β1 expression levels in lung tissues in each group were determined by real-time PCR. **(B)** TGF-β1 activity in lung tissues was measured by an ELISA kit. **(C)** TGF-β1 protein expression in lung tissues in each group was measured by western blot analysis. **(D)** The densitometry values of the proteins were normalized to those of β-actin. All data represent the mean ± SEM of three independent experiments performed in triplicate. Statistical analysis was performed by one-way ANOVA and Turkey’s multiple-comparison test; compared with control group, ^##^*P* < 0.01; compared with BLM group, ^∗^*P* < 0.05, ^∗∗^*P* < 0.01.

Since Smad2/3 phosphorylation by the activated TGF-β1 receptor is a major regulator of the initiation of TGF-β signal transduction, we examined Smad2 and Smad3 activation in the lungs of BLM-treated mice. Smad2 and Smad3 phosphorylation was increased in the BLM group compared with the control group, as confirmed by western blot analysis with antibodies to phosphorylated Smad2 and Smad3 (**Figure 6**). Treatment with GHK markedly inhibited these BLM-activated signaling molecules in a dose-dependent manner. These observations suggest that GHK protects mice against BLM-induced pulmonary fibrosis at least in part by inhibiting the TGF-β/Smad2/3 pathway.

**FIGURE 6:** Effects of GHK on the Smad2/3 signaling pathway in the lung tissues of mice with BLM-induced fibrosis. **(A)** p-Smad2/3 protein expression in lung tissues in each group was measured by western blot analysis. **(B,C)** The densitometry values of the proteins were normalized to those of total Smad2/3. All data represent the mean ± SEM of three independent experiments performed in triplicate. Statistical analysis was performed by one-way ANOVA and Turkey’s multiple-comparison test; compared with control group, ^##^*P* < 0.01; compared with BLM group, ^∗^*P* < 0.05, ^∗∗^*P* < 0.01.

### GHK Reduces the Expression of IGF-1 in Bleomycin-Induced Pulmonary Fibrosis

It has been proved that IGF-1 plays important role in the regulation of cytokines in fibrosis, thus we measured the expression of IGF-1 in BLM-induced pulmonary fibrosis and the effect of GHK on IGF-1 expression. Our findings showed that BLM stimulation could increase the expression of IGF-1 in lung tissue while GHK treatment could reverse this increase in the BLM-induced pulmonary fibrosis (**Figure 7**).

**FIGURE 7:** Effects of GHK on IGF 1/2 expression in lung tissues in mice with BLM-induced fibrosis. **(A)** IGF 1/2 expression, as measured by western blot analysis, in lung tissues in each group. **(B)** The densitometry values for the proteins were normalized to those of β-actin. All data represent the mean ± SEM of three independent experiments performed in triplicate. Statistical analysis was performed by one-way ANOVA and Turkey’s multiple-comparison test; compared with control group, ^##^*P* < 0.01; compared with BLM group, ^∗^*P* < 0.05, ^∗∗^*P* < 0.01.

## Discussion

Bleomycin-induced pulmonary fibrosis is characterized by inflammation and fibrosis in lung tissue and is the most commonly used mouse model for evaluating the anti-fibrotic effects of candidate drug compounds. GHK has been confirmed to ameliorate fibrosis-induced tissue injury in rat models of glomerulonephritis (Isaka et al., 1996) and to suppress the production of scar forming proteins by acting at dermal damage sites (Pickart, 2008). Consistent with the findings of other studies, we found that GHK protected the lungs from BLM-induced fibrosis, inflammation and EMT through the IGF-1 and TGF-β/Smad2/3 signaling pathways. Our experiments showed that treatment with GHK clearly inhibited BLM-induced chronic lung inflammation and fibrosis and reversed BLM-induced weight loss and increases in the lung W/D weight ratio. Furthermore, GHK treatment remarkably repressed the release of inflammatory cytokines, including TNF-α and IL-6, in the lung. BLM-induced EMT was attenuated by treatment with GHK. To our knowledge, this is the first study to employ GHK as an anti-fibrosis treatment in pulmonary fibrosis. The effect of the GHK on bleomybin-induced pulmonary fibrosis has been summarized in **Figure 8**. Our experiment demonstrated the effects of GHK on pulmonary fibrosis and provided new evidence regarding the potential therapeutic effects of GHK on fibrotic diseases.

**FIGURE 8:** Summary of the effects of GHK on pulmonary fibrosis. GHK exerts anti-fibrotic effects through the IGF-1 and TGFβ1/Smad2/3 signaling pathway and attenuates collagen deposition, the inflammatory response and EMT.

Gly-His-Lys was first applied in research regarding wound healing and dermal repair (Gruchlik et al., 2012, 2014). GHK enhances dermal wound healing and stimulates skin renewal by degranulating platelet release growth factors (such as TGF-β), which mobilize immune cells and attract them to sites of injury (Gruchlik et al., 2014). In normal human fibroblasts, GHK reduces the secretion of TGF-β and inflammatory cytokines, such as TNF-α and IL-6, to relieve skin inflammation and prevent the formation of hypertrophic scars (Gruchlik et al., 2012). When treated with GHK, lung fibroblasts from patients with COPD displayed decreased TGF-β activity, indicating that GHK corrects defects in collagen gel remodeling in patients with COPD (Campbell et al., 2012). GHK is naturally occurring, non-toxic, and readily forms complexes with copper, improving the bioavailability of GHK. Comparing to GHK, GHK copper (II)-chelated form (GHK-Cu) also showed similar or even better effects on wound healing, improvement in the success of transplanted skin, and acute lung injury under some conditions (Arul et al., 2007; Pickart et al., 2015; Park et al., 2016). These findings support the idea that GHK improves tissue regeneration and anti-fibrotic processes. In this study, we demonstrated the protective effects of GHK against pulmonary fibrosis. Specifically, we demonstrated the anti-inflammatory and anti-fibrotic effects of GHK. In order to gain the maximum benefit of GHK and GHK-Cu, optimizing the administration way should be paid attention to. It is found that nanoscaled liposomes encapsulating GHK-Cu promoted human umbilical vein endothelial cells proliferation with a 33.1% increase rate (Wang et al., 2017). Another research has discovered the GHK-Cu(2+)-loaded Zn-pectinate microparticles in form of hydroxypropyl cellulose (HPC) compression-coated tablets for colon delivery of GHK which indicated the possibility of GHK for internal use (Ugurlu et al., 2011). But when the pulmonary diseases are concerned, the tropical and effective delivery way should be explored and tested in future.

The transitions of alveolar epithelial cells into fibroblast and fibroblasts into myofibroblasts are crucial to the pathogenesis of pulmonary fibrosis. EMT involves a distinct integrin-sensing system that activates TGF-β1 (Marmai et al., 2011). Our results showed that EMT occurred in BLM-induced fibrosis, a phenomenon reflected by elevations in the protein levels of α-SMA, fibronectin, and vimentin and decreases in the protein levels of E-cadherin. Treatment with GHK attenuated the transition of alveolar epithelial cells into fibroblasts. These findings demonstrate that GHK prevents the transition of epithelial cells into collagen-producing myofibroblasts through the TGF-β1 pathway.

The TGF-β1/Smads signaling pathway is known to play a predominant role in the pathological process of fibrosis and occurs as a result of receptor–ligand interactions resulting in the rapid phosphorylation and nuclear translocation of Smad2 and Smad3 (Nakao et al., 1997; Hu et al., 2003). Many experimental studies have reported that the inhibition of TGF-β by anti-TGF-β antibodies (Giri et al., 1993), TGF-β soluble receptors (Kolb et al., 2001), or TGF-β peptide inhibitors (Arribillaga et al., 2011) has a protective effect against the development of pulmonary fibrosis. Zhao et al. (2002) demonstrated that Smad3 deficiency also attenuates BLM-induced pulmonary fibrosis in mice. Furthermore, a recent study showed that decreasing TGF-β1-induced Smad2 protein expression had clear anti-fibrotic effects (Jin et al., 2015). Our study showed that TGF-β1and p-Smad2/3 levels were apparently increased after intratracheal BLM instillation for 21 days and that GHK attenuated these changes. The effects of GHK on the expression levels of these proteins paralleled its effects on BLM-induced lung histopathological changes. In the present study, GHK treatment effectively inhibited BLM-induced TGF-β1 and Smad2/Smad3 expression, results consistent with those of previous studies showing that GHK has inhibitory effects on TGF-β1expression (Isaka et al., 1996; Simeon et al., 2000; Pickart, 2008). Taken together, our observations indicate that the anti-fibrotic effects of GHK may be due to the inhibition of the TGF-β/Smads pathway. Our study is the first to reveal that GHK may protect against pulmonary fibrosis by affecting the TGF-β1/Smads signaling pathway.

Transforming growth factor-β1 production may be controlled at the transcription and translation levels, as well as the levels at which the preformed protein is secreted, and the latent protein is activated (Sullivan et al., 2005). IGF-1, which exerts its main effects through the IGF-1 receptor, is important for the regulation of cytokines in physiological and/or pathological processes, such as cellular proliferation, differentiation (De Meyts et al., 1994; Cohen, 2006a,b), and fibrosis (Hinz et al., 2001; Cohen, 2006b; Hinz, 2007; Gruchlik et al., 2014). IGF-1 mRNA and protein levels were up-regulated in the murine BLM lung fibrosis model compared with the control group (Maeda et al., 1996; Choi et al., 2009). These findings show that stimulating fibroblasts with IGF-1 enabled fibroblasts to differentiate into a myofibroblast phenotype in a soft matrix environment and thus stimulate collagen deposition (Hung et al., 2013). In this study, we found that IGF-1 protein levels increased after the intratracheal instillation of BLM for 21 days, suggesting that IGF-1 was involved in pulmonary fibrosis and tissue injury. These changes were suppressed by GHK treatment. In previous studies, IGF-1 treatment caused the substantial induction of TGF-β1 mRNA and protein expression, resulting in the formation of a hypertrophic scar (Ghahary et al., 1998; Wang et al., 2000). In a previous study, alveolar macrophage released IGF-1 and TGF-β in IPF and participated in both inflammation and fibrosis (Cao et al., 2000). Taken together, these findings show that the effects of GHK on pulmonary fibrosis may be mediated by crosstalk between IGF-1and TGF-β1/Smads signaling pathway activation.

There were several limitations to our study. We concentrated on the anti-fibrotic effects of GHK, which attenuated IPF injury by inhibiting the IGF-1-mediated TGF-β1/Smads signaling pathway. We did not block IGF-1 to confirm our findings, we did not compare the difference in efficacy between GHK and GHK-Cu, ether. So we cannot confirm whether GHK-Cu is better than GHK in protective effects on BLM induced lung fibrosis of mice model. Besides, due to the limited application of the GHK in the animal experiment, the dose-response curve has not been covered in our study. So further research regarding this issue is needed.

## Conclusion

Our mouse model suggests that BLM works via mechanisms dependent on IGF-1 to activate the TGF-β1/Smads signaling pathway, leading to pulmonary fibrosis. GHK attenuates BLM-induced pulmonary fibrosis by decreasing the expression of IGF-1 and inhibiting the activation of the TGF-β1/Smads signaling pathway. GHK may thus be a candidate for the treatment of pulmonary fibrosis.

## Author Contributions

Substantial contributions to the conception or design of the work: GH. Acquisition of data for the work: All authors. Analysis of data for the work: X-MZ, G-LW, X-BW, LL, YY, and QZ. Interpretation of data for the work: GH. Drafting the work: X-MZ, GH, and X-BW. Revising it critically for important intellectual content: All authors. Final approval of the version to be published: All authors. Agreement to be accountable for all aspects of the work in ensuring that questions related to the accuracy or integrity of any part of the work are appropriately investigated and resolved: X-MZ, G-LW, X-BW, LL, QZ, YY, Q-YW, JK, GH.

## Conflict of Interest Statement

The authors declare that the research was conducted in the absence of any commercial or financial relationships that could be construed as a potential conflict of interest.

## Abbreviations

ANOVA: analysis of variance
BALF: bronchoalveolar lavage fluid
BLM: bleomycin
COPD: chronic obstructive pulmonary disease
ELISA: enzyme-linked immunosorbent assay
EMT: epithelial mesenchymal transition
GHK: Gly-His-Lys
HE: hematoxylin-eosin
IGF-1: insulin-like growth factor-1
IPF: idiopathic pulmonary fibrosis
MPO: myeloperoxidase
MT: Masson’s trichrome
TGF: transforming growth factor
TNF: tumor necrosis factor
W/D: wet-to-dry
